RETRACTED

# A Review of Intelligent Driving Pedestrian Detection Based on Deep Learning

**DOI:** 10.1155/2021/5410049

**Published:** 2021-07-20

**Authors:** Di Tian, Yi Han, Biyao Wang, Tian Guan, Wei Wei

**Affiliations:** ^1^School of Automobile, Chang'an University, Xi'an, Shaanxi 710064, China; ^2^School of Computer Science and Engineering, Xi'an University of Technology, Xi'an, Shaanxi 710048, China

## Abstract

Pedestrian detection is a specific application of object detection. Compared with general object detection, it shows similarities and unique characteristics. In addition, it has important application value in the fields of intelligent driving and security monitoring. In recent years, with the rapid development of deep learning, pedestrian detection technology has also made great progress. However, there still exists a huge gap between it and human perception. Meanwhile, there are still a lot of problems, and there remains a lot of room for research. Regarding the application of pedestrian detection in intelligent driving technology, it is of necessity to ensure its real-time performance. Additionally, it is necessary to lighten the model while ensuring detection accuracy. This paper first briefly describes the development process of pedestrian detection and then concentrates on summarizing the research results of pedestrian detection technology in the deep learning stage. Subsequently, by summarizing the pedestrian detection dataset and evaluation criteria, the core issues of the current development of pedestrian detection are analyzed. Finally, the next possible development direction of pedestrian detection technology is explained at the end of the paper.

## 1. Introduction

Object detection is a basic problem of machine vision and deep learning, and it lays the basis for the in-depth development of numerous research problems, including instance segmentation [1–3], object tracking and optimization [4–6], trajectory prediction [7], and image reconstruction [8–10]. Pedestrian detection is a specific application of the object detection problem, and it has become one of the research hotspots in recent years. It has important application value in the fields of intelligent driving and security monitoring. Particularly in the field of intelligent driving, due to the particularity of people and the highest safety requirements, it is more important than other types of object detection. In intelligent driving, the camera, lidar [11–13], and wireless sensor network [14–18] jointly perceive the environment and further employ vehicle-mounted computers and cloud computing [19–23] to make decisions and control.  Figure 1 presents the trend of the number of publications in association with pedestrian detection in recent years. Compared with other types of object detection, pedestrian detection puts forward stricter requirements on accuracy and real-time performance, which is of extraordinary significance in the field of intelligent driving. In recent years, large quantities of reviews of general object detection have been published [24–28], but there are few reviews of pedestrian detection, lacking the analysis of its latest developments and discussion of current difficulties. By performing a rough analysis of general object detection, this paper will discuss in-depth pedestrian detection.

RETRACTED

The development of object detection tasks has mainly experienced two major stages, respectively, the traditional object detection period and the detection period based on deep learning. As early as 2001, P. Viola and M. Jones proposed the famous VJ detector [29]. It combines a variety of important technologies such as “integral image,” which significantly improves the detection efficiency and detection capabilities and realizes the real-time detection of fixed object for the first time, strongly promoting the development of the object detection field. In particular, in 2005, Dalal and Triggs proposed the Histogram of Oriented Gradients (HOG) feature descriptors [30], which designed the HOG descriptors to be calculated on a dense uniformly spaced cell grid and adopted overlapping local contrast to normalize in order to improve the accuracy. Although HOG can be used to detect various object classes, its main research goal is to solve the problem of pedestrian detection. The proposed method has achieved a very high accuracy rate, which strongly demonstrates the effectiveness of this algorithm. Subsequently, in order to promote the development of the field of pedestrian detection, the INRIA pedestrian dataset, which is still widely used, was published. Later in 2008, Felzenszwalb proposed the DPM detection algorithm [31], which can divide pedestrian into different parts for training and learning as well as treating them as a collection of different parts detection during classification. Under this kind of thinking, the algorithm and its improved algorithm have continuously obtained the best detection results for several years, reaching the relative peak of traditional detection algorithms. Additionally, there are scholars who study general computer vision methods, which can improve various computer vision problems [32–37].

The implementation process of the traditional object detection method is similar to the VJ detector. It mainly extracts object features through artificial design (such as HOG, Haar, and SIFT) and new feature extraction methods [38, 39] and further uses SVM, DT [40], and other classifiers for recognition and detection. Before the detection, the image is often preprocessed to enhance the image quality [41–43]. In the detection process, sliding window processing is usually performed on the image to predict the object. At that time, the best detection performance is achieved. However, because the sliding window method traverses all possible positions and size ratios, it places high requirements on the computing power of the computer. In addition, the hand-designed feature expression ability is weak, contributing to a poor overall detection effect. In 2014, Girshick et al. proposed the RCNN algorithm [44] for feature extraction using CNN. This algorithm vigorously stimulated the development of object detection tasks and advanced it to the development stage of deep learning. In general, deep learning can use the gradient descent method to automatically optimize model parameters [45]. Various object detection tasks have achieved leap-forward progress. Later, some optimization methods in association with neural networks appeared [46–48]. At present, neural networks have a wide range of applications [49–53]. The development process of pedestrian detection is displayed in Figure 2.

RETRACTED

The rest of the work is arranged as follows. In the second part, the current mainstream pedestrian detection algorithms are summarized. In the third part, the commonly used datasets and evaluation methods in the pedestrian detection field are presented. In the fourth part, the occlusion problem and the multiscale problem that affect the pedestrian detection effect are analyzed in detail. The full text is summarized and prospected in the fifth part.

## 2. Pedestrian Detection Method Based on Deep Learning

Since Girshick et al. proposed RCNN in 2014, the task of pedestrian detection has officially entered the deep learning stage. In general, detection methods based on deep learning mainly consist of two categories. One is a two-stage processing method. Firstly, regional suggestion boxes for possible object are generated, and then further predictions are made on these suggestion boxes. The other is a one-stage processing method, which directly returns the object area on the feature map and gives the final prediction result. The following part summarizes the specific applications of these two detection frameworks in pedestrian detection.

### 2.1. Two-Stage Detection Framework

The two-stage detection framework is mainly divided into two stages: region suggestion and object detection. First, a series of region suggestion boxes are proposed on the image to be inspected. Then, object detection is further conducted. The RCNN detection framework proposed by R. Girshick in 2014 first uses selective search [54] to generate a region suggestion box on the image, then uses CNN for feature extraction, further trains the SVM classifier and bounding-box regression, and finally predicts the result. Although the use of CNN for feature extraction greatly improves the detection effect, it also encounters many problems, such as cumbersome training process and long detection time. Subsequently, improved Fast RCNN [55] and Faster RCNN [56] algorithms are proposed to address the above problems. Faster RCNN completes the end-to-end detection process. First, the RPN algorithm is proposed to replace the selective search for regional recommendation, which greatly reduces the time consumed by regional recommendations. In addition, shared features help avoid repeated feature calculations, the detection accuracy on the VOC07 dataset [57, 58] reaches 73.2%, and the detection accuracy on the COCO dataset [59] reaches 42.7%. The framework diagram of the Faster RCNN series of algorithms is shown in Figure 3.

RETRACTED

In 2015, Cai et al. deduced that the Comp ACT algorithm [60] not only optimizes classification risk but also better combines feature extraction and classifier function, which plays an important role in promoting pedestrian classification at different scales. In 2016, Dai et al. made a series of improvements based on Faster RCNN and proposed RFCN [61]. RFCN integrates location information into the pooling layer, enhances location sensitivity, and improves the processing results of pedestrian detection problems that are more sensitive to location information. Compared with Faster RCNN, the introduction of FCN achieves more network parameters and feature sharing, reduces the amount of repetition in the network, and improves the running speed. In 2017, the Mask RCNN proposed by Kaiming He et al. adds a convolutional layer after the pooling layer to perform mask prediction tasks. This structure can complete tasks such as pedestrian detection and pedestrian segmentation and separate pedestrians from the background. At the same time, the result can be further used for human body gesture recognition.

In 2017, Lin et al. proposed FPN [62] based on Faster RCNN. Before that, most of the detectors were detected at the top of the network. Although it has good semantic information for category detection, it is not conducive to pedestrian positioning due to the small feature map. FPN proposes a top-down prediction structure and builds high-level semantic information on the entire convolution structure, making pedestrian detection greatly improved.

In 2018, Li et al. proposed SAF RCNN based on the perception theory [63], which effectively improved the performance of pedestrian detection of different scales.

RETRACTED

Among the two-stage detection methods based on deep learning mentioned above, the RCNN series methods (RCNN [44], Fast RCNN [55], and Faster RCNN [56]) are the earliest ones proposed in recent years. The RCNN series method is a general object detection method, which is not specially optimized for a typical category and can be used in various object detection tasks. The main constraints on the performance of RCNN and Fast RCNN are repeated convolution calculations and region proposal networks, which have been improved in Faster RCNN and achieved the best results at the time. The Comp ACT algorithm [60] introduced above is mainly used in the field of pedestrian detection. This algorithm can improve the processing capacity of pedestrian detection and can be extended to other object detection problems to a certain extent. The RFCN [61] algorithm is mainly proposed for general object detection, and it can also achieve good results in specific pedestrian detection areas. Mask RCNN [3] is an improvement based on Faster RCNN. It is a solution proposed for general object detection, and it also has a good effect in the field of pedestrian detection. The FPN [62] algorithm constructs a feature pyramid network, which greatly improves the general object detection and pedestrian detection problems. The SAF RCNN [64] algorithm is mainly used in the field of pedestrian detection in natural scenes. It can also improve the general object detection ability, but because the object scale change is more common in the field of pedestrian detection, the improvement in general object detection is limited.  Table 1 summarizes the calculation speeds of the two-stage detection methods mentioned above.

There are two parts in the two-stage pedestrian detection framework: region suggestion and classification. Researchers can improve the detection effect by proposing different preselection box generation algorithms and feature extraction algorithms or improve the detection results by enhancing the prediction part. Although the overall framework is more cumbersome than the one-stage framework, it has better robustness and accuracy overall.

### 2.2. One-Stage Detection Framework

Compared with the two-stage detection framework, the one-stage detection framework removes the preselection box generation algorithm and directly predicts the object center and object bounding box by setting a series of anchors on the feature map. In 2015, Redmon et al. proposed the first single-stage detector YOLO [65] in the deep learning era. The idea of this detector is shown in Figure 4. It applies a single neural network to the entire image and divides the image into multiple regions. This mode greatly improves the detection speed while predicting the bounding box and probability of each region simultaneously. In the task of pedestrian detection, especially in the pedestrian detection of intelligent driving technology, the detection speed is particularly important [66]. Only high-speed detection can avoid a series of hazards. The one-stage detection framework provides the possibility for this.

RETRACTED

Compared with the two-stage detector, the positioning accuracy of YOLO has decreased, and because it only predicts a limited number of objects at a prediction anchor, the detection effect for small objects and group objects is poor. In response to the above problems, J. Redmon proposed YOLOv2 [67] and YOLOv3 [68]. They were optimized for the above problems, which not only greatly improved the detection accuracy of the one-stage detector but also achieved a relative balance between speed and accuracy. Particularly for YOLOv3, three prediction channels are used to improve the effect of multiscale prediction in pedestrian detection. The structural frame diagram of YOLOv3 is displayed in Figure 5.

In 2016, Liu et al. further proposed an SSD one-stage detection framework [69]. Unlike YOLO, the SSD algorithm outputs feature layers of different sizes through multilayer mapping in the convolutional layer to detect multiscale objects. In particular, the detection effect of small objects is improved.

In 2017, Lin et al. proposed the RetinaNet detector [70]. In response to the poor detection effect of the one-stage detector, a new loss function is introduced in it, so that the detector pays more attention to the difficulty in classifying samples during the training process and solves the problem of unbalanced samples in the work of the one-stage detector. Overall, the single-stage detector can improve its detection accuracy while maintaining a high detection speed. In 2018, Liu et al. put forward an efficient one-stage pedestrian detection architecture ALFnet [71], which mainly uses the continuously increasing IOU threshold to train multiple positioning modules. It can improve the detection accuracy of pedestrian detection. It can achieve the same detection speed as SSD and the same detection accuracy as Faster RCNN; at that time, the most advanced performance was achieved on the CityPersons dataset and the Caltech dataset. In 2019, Zheng et al. proposed DIOU Loss and CIOU Loss [72] to optimize the previous loss function. Compared with the previous object box regression loss, it considers the overlap area, center point distance, and aspect ratio. The bounding box considering the distance loss has faster convergence speed and higher convergence accuracy, which improves the detection accuracy of the object detection framework.

RETRACTED

In 2020, Alexey Bochkovskiy proposed YOLOv4 [73]. Based on the advantages of multiple detection frameworks, Backbone partially uses the CSPNet structure [74] proposed by Wang et al. in 2020. The schematic diagram of applying CSP to ResNet is shown in Figure 6, which adds a path to each cycle block. In the neck part, the feature fusion is performed by adding the SPP structure [75] and the PAN structure [76]. In addition, the advantages of clustering [77] are used to generate the predicted frame size. The SPP structure can help the network integrate the features of different scales, and the PAN structure integrates the features obtained from different layers. Finally, YOLOv4 obtains 65.7% (AP50) detection accuracy and 65FPS detection speed on the coco dataset, achieving the best balance between the current detection frame speed and accuracy. In addition, some scholars study the application of object detection to slam so as to promote the development of related technologies [78]. So far, pedestrian detection algorithms have mostly focused on the two-stage network framework. However, pedestrian detection in intelligent driving technology has high requirements for real-time performance. With the breakthroughs in accuracy and real-time performance of frameworks such as YOLOv4, pedestrian detection technology in the future will focus more on the single-stage detection framework. Beyond that, these algorithms have also laid a solid foundation for the application of pedestrian detection in intelligent driving.

Among the above-mentioned one-stage detection methods based on deep learning, the YOLO series methods (YOLOv1 [65], YOLOv2 [67], YOLOv3 [68], and YOLOv4 [73]) are the earliest ones proposed in recent years. The algorithms of the YOLO series can be used in various object detection tasks. Due to the reason that only a limited number of objects are predicted in one anchor, it often causes missed detection in the scene of crowded pedestrians, so the performance of the algorithm will be reduced in the crowded scene. However, the high detection speed of such algorithms provides the possibility for the application of pedestrian detection technology in the field of intelligent driving. The SSD [69] algorithm mentioned above is proposed for general object detection, which can improve the problem of multiscale detection in pedestrian detection. The RetinaNet [70] detector introduces a new loss function, which can improve the detection accuracy in the general object detection field. The ALFnet [71] algorithm is mainly used for pedestrian detection. Due to the effective improvement of the task of pedestrian detection, it can be extended to general object detection to a certain extent. The CIOU Loss [72] algorithm researches the boundary regression problem in object detection, which effectively improves the detection effect of various objects.  Table 2 summarizes the calculation speeds of the one-stage detection methods mentioned above.

RETRACTED

### 2.3. Backbone

The pedestrian detection algorithms are different. However, in the deep learning stage, the first is to use the convolutional neural network to process the image to obtain the deep feature map and then perform various subsequent processing. This part obtains the convolutional neural network of the feature map called the “Backbone” of the entire algorithm. Backbone can decisively influence the effect of the network. This section will review this content.

#### 2.3.1. VGGNet

After AlexNet [79] achieves excellent results in the ImageNet competition, the VGGNet [80] proposed by Simonyan in 2014 improves the convolutional neural network, uses a smaller convolution kernel and a deeper network structure, and achieves better results.

#### 2.3.2. INception

In the process of extracting features of the convolutional neural network, increasing the depth and width of the network can improve the performance of the network. Nonetheless, doing so will also lead to a substantial increase in the number of parameters, and it is prone to overfitting. Inception [81], proposed in 2014, solves this problem better. It uses three convolution kernels of different sizes for convolution calculations and then cascades these parts to enter the next layer. Later, the improved *v*2, *v*3, and *v*4 versions [82–84] are proposed.

#### 2.3.3. ResNet

Based on VGGNet and Inception, He et al. proposed ResNet [85] in 2015, solving the problem of gradient disappearance and gradient update difficulty. Since then, ResNet has been generally used as Backbone for various classification, detection, and segmentation tasks. The main idea is to introduce a residual block, let the convolutional network learn the residual mapping, and make the network optimization easier.

#### 2.3.4. DenseNet

In 2017, DenseNet [86] maximized the information exchange between the front and rear layers based on ResNet. By establishing dense connections between all the front layers and all the back layers, it realizes the multiplexing of features in the channel dimension. This structure can achieve better performance than ResNet with fewer parameters and calculations.

#### 2.3.5. FPN

In order to enhance semantics, traditional object detection models usually only perform follow-up operations on the last feature layer, but the final feature map often has less detailed information, making the detection of small objects more difficult. In 2017, the FPN method merged the features of different layers, which better improves the multiscale detection problem. The overall architecture of FPN mainly consists of four parts: bottom-up network, top-down network, horizontal connection, and convolution.

RETRACTED

#### 2.3.6. DetNet

DetNet [87] introduces the hole convolution, which increases the receptive field, obtains a larger feature map size, and makes the model have a larger receptive field and higher resolution. At the same time, the detection of large objects and small objects is taken into account. It is especially suitable for inspection tasks. The structure diagram is shown in Figure 7.

## 3. Dataset and Evaluation Method

### 3.1. Dataset

The dataset is the basis of the pedestrian detection task. It not only is a data source for researchers to conduct experimental tests but also provides the same data basis for the performance comparison of different algorithms. Measuring the quality of a dataset includes the amount of data and the quality of labeled information. The richness of the dataset determines the robustness of the detector to a certain extent. Compared with general object detection tasks, pedestrian detection has its own unique characteristics. Common pedestrian detection datasets now include Caltech [88], KITTI [89], CityPersons [90], TUD [91], and EuroCity [92]. In addition, the current common dataset in the object detection field is COCO. The relevant information of these datasets is shown in Table 3. According to the different content of each dataset, it has its own characteristics. Among them, the Caltech, KITTI, and CityPersons datasets have more complete labeling information and are more widely used. The images in these three datasets are shown in Figure 8. Here is a brief introduction to these datasets.

#### 3.1.1. CALTECH

Caltech is currently the largest pedestrian detection dataset, which includes 350,000 pedestrian bounding boxes marked in 250,000 frames of images, and the occlusion and the corresponding time are also marked.

#### 3.1.2. KITTI

The KITTI dataset is currently the largest computer vision algorithm evaluation dataset in autonomous driving scenarios. This dataset is used to evaluate the performance of computer vision technologies such as stereo, optical flow, visual odometry, 3D object detection, and 3D tracking in a vehicle environment. KITTI contains real image data collected from scenes such as urban, villages, and highways. There are up to 15 cars and 30 pedestrians in each image, with various degrees of occlusion and truncation.

RETRACTED

#### 3.1.3. CityPersons

The Cityscapes city dataset contains street scenes from 50 different cities recorded from a set of different stereo video sequences and the pixel-level annotation of the image. It mainly labels the data of pedestrians on urban roads to obtain a pedestrian detection dataset.

### 3.2. Evaluation Method

The detection ability of the pedestrian detector is mainly reflected by the corresponding evaluation index, and an excellent evaluation method can objectively reflect the detection ability of the detector. Generally, the detector is trained through the train set of the dataset, and then the detector is evaluated through the test set.

At present, the most commonly used evaluation for object detection is Average Precision (AP). Generally, the performance of the model is dynamically evaluated by drawing a P-R curve, where the horizontal coordinate is the recall rate and the vertical coordinate is the accuracy rate. In order to compare the performance of all object categories in multiclass detection, the mean Average Precision (mAP) of all object categories is usually used as the final metric of performance. In order to measure the accuracy of object positioning, Intersection over Union (IoU) is used to check whether the overlap ratio between the prediction box and the ground truth box is greater than a predefined threshold, which is generally defined as 0.5. If it is greater than this value, the object will be recognized as successfully detected; otherwise, it will be defined as missed. After 2014, due to the widespread use of COCO datasets, researchers began to pay more attention to accuracy. In COCO, a fixed IoU threshold is not used. Instead, take the average of multiple IoU thresholds between 0.5 (coarse positioning) and 0.95 (perfect positioning). This metric change promotes more accurate object positioning.

In addition, some scholars found in their research that only using the precision-recall curve cannot accurately express the effectiveness. Piotr proposed the MR-FPPI curve in 2012, where MR represents the missed detection rate and FPPI represents the number of false detections per image. This evaluation method is commonly used in the field of pedestrian detection.

In the Caltech dataset, the detection results of some of the most advanced algorithms for pedestrian detection in overall data, far scale data, and heavy occlusion data are shown in Tables 4–6.

## 4. General Issues

At present, the detection ability of mainstream detectors for general images has been developed by leaps and bounds, especially the images of short distances and large objects for which very good detection results can be obtained. Currently, the main restriction of the further development of pedestrian detection lies in the detection ability for low-quality images, including the key issues such as multiscale and occlusion. This section will analyze these issues.

RETRACTED

### 4.1. Occlusion Issue

Crowding and occlusion between objects are the common difficulties in pedestrian detection [98], as shown in Figure 9, causing the loss of information of the object, and invisibility of part of the area, which is likely to cause false or missed detection by the detector.

Compared with general object detection, occlusion is more likely to happen in pedestrian detection because group movement behaviors are prone to occur in pedestrians, which is also a major obstacle limiting the application of pedestrian detection in autonomous driving tasks. In the CityPersons dataset, the proportion of pedestrian occlusion is shown in Table 7, and the occlusion between pedestrians has a serious impact on the accuracy of pedestrian positioning, which is more sensitive to the NMS threshold, thereby easily suppressing the candidate frames of similar pedestrians.

Due to the lack of information for pedestrians under occlusion, researchers used variable part models to solve the related problems at the beginning. Although the detection results have been improved to a certain extent, the amount of model calculations has increased sharply [99–101]. To break through the limitations of multicomponent detectors, Ouyang et al. integrated detectors with occlusion of different degrees [102], thus effectively shortening the detection time, and in the further research integrated the part model into the neural network to improve the detection effect. Though an effective method is available to improve the effect of pedestrian detection under occlusion based on partial model-assisted global detection [103], it is at the price of increased computational cost and reduced detection speed. Therefore, one of the main research directions of this method is to improve the recognition rate of the detector for blocked pedestrians while maintaining the detection speed.

Similar to the part model method that uses a series of component detectors to merge with each other, another solution takes the advantages of the attention mechanism [104] to focus on key parts of pedestrians for occlusion detection. As a model, SSA-CNN [105] uses the attention mechanism to perform occlusion detection, thereby effectively improving the detection effect. In addition, some methods such as SDS-RCNN use semantic segmentation to deal with the occlusion problems, in this manner to make the generated features more focused on pedestrians, locate possible pedestrian areas, and have CNN paying attention to possible pedestrian occlusion parts. The main idea of this method is to quickly locate pedestrians and focus on the characteristics of the pedestrian's location. The SDS-RCNN framework is shown in Figure 10.

RETRACTED

In addition to the above-mentioned methods used to solve the occlusion problem in pedestrian detection, some scholars focused on postprocessing. Liu et al. proposed an Adaptive NMS [106] method to solve the problem of sensitivity to the NMS threshold in pedestrian detection, thereby effectively improving the detection efficiency. In addition, Wang et al. designed a new repulsive loss function RepLoss [107] to reduce the mutual influence between objects, which effectively alleviates the detection effect in the case of pedestrian occlusion. Zhang et al. proposed that OR-CNN [108] can improve the loss function and ROI Pooling based on Faster RCNN and introduced the idea of part-based which effectively alleviates the problem of pedestrian occlusion.

At present, the processing of pedestrian detection and occlusion problems has gradually shifted to the CNN itself and from the improvement of the overall network architecture to the improvement of each processing stage.

Among the algorithms introduced above, the algorithms [99–101] are all early methods based on deformable parts, which are mainly used for pedestrian detection. This type of method is not universal and needs to be designed for specific detection objects. Similarly, the algorithm [102, 103] is also designed for the problem of pedestrian occlusion, and it is difficult to generalize to the field of general object detection. SDS-RCNN [94] and SSA-CNN [105] are mainly designed for pedestrian detection to improve the effect of pedestrian detection. Adaptive NMS [106] is mainly designed for the crowding problem in pedestrian detection. This algorithm can be extended to the general object detection field to a certain extent, reducing the error of common use NMS algorithms. Similar to [106], RepLoss [107] and OR-CNN [108] are mainly designed for pedestrian detection and can be extended to general object detection to a certain extent. However, because these algorithms are specifically designed for pedestrian detection, the improvement in general object detection is limited. The calculation speeds of some of the above algorithms are summarized in Table 8.

### 4.2. Multiscale Issue

The traditional convolutional neural network adopts a single-line structure, and the shallow feature map has a larger area and contains more detailed information, making it suitable for detecting small objects. The deep feature map, which has a small area and only contains semantic information, is suitable for the detection of large objects. Generally, convolutional neural networks present the problem of multiscale detection of large and small objects, which has not been well solved [109]. The multiscale pedestrian image is illustrated in Figure 11. For small object detection, reducing the downsampling rate of the network, which is the simplest way to improve detection capability, can increase the detailed information on the feature map. Besides, a hole convolution can be used to increase the receptive field of the subsequent layer when the downsampling rate is reduced. This convolution method cannot guarantee that the receptive field after the modification is consistent with that before the modification but can minimize the degree of change as much as possible. Moreover, many methods [110–112] have been proposed to solve this problem.

RETRACTED

With the purpose of improving the multiscale detection capability, several different image input scales can be set in the training phase. During training, one is randomly selected from multiple scales, and the picture is scaled to this scale and input into the network, contributing to an increase in the robustness of the network without raising the amount of calculation. Song et al. proposed the TLL method [113], which improved the detection results by establishing human body model information at different scales. However, Zhang et al. have effectively reduced the missed detection rate by further investigating the label information [114].

With the increase in the number of layers, the traditional convolutional network will enlarge the receptive field and enrich the semantic information while causing severe loss of the information of the small object at the output of the network. Its small object detection ability is very poor. The idea of feature fusion [115–120] is to combine deep and shallow layers, fuse the features of the two, and complement each other's advantages, so as to improve detection performance. RPN has this effect; however, the improvement of pedestrian detection effect for small objects is limited. Li et al. and Cai et al. proposed SAF RCNN and MS-CNN, respectively, to deal with scale changes. Besides, SSD also enhances the detection effect by combining different feature layers for feature fusion. Generally, the key to multiscale detection is whether the feature extraction stage can extract pedestrian features at various scales.

The researcher proposing the TridentNet network [121] changed the number of holes in the last convolutional layer by analyzing the influence of different sizes of receptive fields on the detection results. He parallelized three different receptive fields and compared the previous basic network results. The detection results demonstrate a significant improvement in accuracy. The network diagram is illustrated in Figure 12.

RETRACTED

In pedestrian detection, the current effective methods for solving multiscale problems include reducing the downsampling rate and convolution of holes, multiscale training MST, feature fusion, and TridentNet. The core idea is to obtain more general detection capabilities at different scales by fully excavating the feature information of different scale features.

Among the algorithms introduced above, the algorithms [110–112] are all designed for pedestrian detection, and part of their content can be extended to general object detection. Similarly, the algorithms [113, 114] are also designed to solve the problem of pedestrian detection and are used to improve the performance of pedestrian detection at different scales. Both MS-CNN [95] and TridentNet [121] are designed for general object detection, and good results can also be obtained in pedestrian detection technology. Compared with other object detection tasks, object scale changes are more common in the field of pedestrian detection, so the algorithm mentioned above can effectively change the effect of pedestrian detection. The calculation speeds of some of the above algorithms are summarized in Table 9.

## 5. Discussion

Object detection is one of the four basic tasks of computer vision, and it is a current research hotspot. The main purpose of this task is to detect specific object instances (“cats,” “dogs,” etc.) from a given image. As a typical object detection task, pedestrian detection is consistent with the general object detection task, which is to detect pedestrians in a given image. In recent years, with the continuous development of deep learning [122, 123], object detection has made great progress, especially the wide application of multicategory datasets such as COCO. Most researches focus on general object detection. As a typical object detection task, pedestrian detection has a special position in fields such as intelligent driving, and it is directly related to driving safety and pedestrian safety. At present, due to the widespread attention of general object detection, there are few reviews in the field of pedestrian detection. For example, references [24, 27] gave a full introduction to general object detection in recent years but did not conduct a detailed analysis of pedestrian detection. Reference [124] mainly discusses the problem of pedestrian detection in far-infrared video and does not involve pedestrian detection technology in natural images. References [88, 114, 125, 126] did not discuss the research progress in the past two years due to time constraints and rarely involved the current research focus on deep learning techniques. Reference [127] mainly discusses Human Detection technology and does not make detailed analysis for pedestrian detection.

RETRACTED

Based on the general analysis of general object detection, this paper makes an in-depth discussion on pedestrian detection problems. The main contributions of this paper are as follows: (1) The pedestrian detection algorithm based on deep learning proposed in recent years is introduced in detail, and its advantages and disadvantages are analyzed. (2) It introduces the common use datasets and evaluation metrics for pedestrian detection. (3) The main issues that limit the performance of pedestrian detection in areas such as intelligent driving are discussed in detail. (4) It explains the future development direction of pedestrian detection. However, this paper does not involve the introduction of pedestrian detection in special scenarios (night, rain, snow, fog, etc.), which is also the direction of future work.

The pedestrian detection technology described in this review is mainly solved by visual methods based on machine learning technology, which is also the current mainstream solution. However, this solution has certain constraints. Although vision-based image processing technology has made great progress, this method has a higher demand for the external environment (light, weather, etc.). On this basis, some people have paid attention to the research of infrared images and made some progress. However, the lack of infrared image datasets limits its development to a certain extent, and it is still sensitive to factors such as occlusion. Vision-based detection technology has its inherent constraints. How to use multisensor fusion technology to improve the effect of pedestrian detection technology in practical applications such as intelligent driving is a major development direction at present. In addition, although the traditional machine learning technology has fast detection speed and low hardware platform requirements, it can no longer meet the current application requirements due to its low detection accuracy. Although the deep learning technology in machine learning technology has made great progress in recent years, the computing model is often large and has high requirements on the hardware platform. It is more difficult to deploy on the mobile terminal with less computing resources such as smart cars. This is also a major factor affecting the development of deep learning technology.

## 6. Conclusions

Pedestrian detection is an important problem of computer vision. Compared with general object detection, it has important research value in the field of intelligent driving. It has similarities and differences with general object detection. This review first introduces the content of general object detection, then analyzes the development of pedestrian detection, and elaborates on the common datasets and main problems faced by pedestrian detection. Although the pedestrian detection technology has made great progress from the original traditional machine learning to the current neural network, there is still a huge gap with human vision. In addition, lightweight network is also a research core. How to deploy it to the mobile terminal without affecting performance directly affects its application in intelligent driving. This review believes that the future development direction of pedestrian detection technology is as follows:

1. The above-mentioned multiscale issues and occlusion issues are the core issues affecting pedestrian detection. Among them, the multiscale issue requires that pedestrians of different sizes can be accurately detected at the same time, which puts higher requirements on the feature extraction network. The occlusion issue requires accurate detection of pedestrian parts and puts forward higher requirements on the recognition algorithm. The improvement of these issues can directly improve the effect of pedestrian detection in complex scenes, which is an important way to improve the ability of pedestrian detectors.
2. Although the current detection network has made great progress, the hardware requirements are often high. Therefore, how to lightweight the network while maintaining the detection performance is an important issue in practical applications. This is also an important direction for future development.
3. At present, the general pedestrian detection still uses a single pedestrian as the object and does not consider the relationship with other objects in the environment. Considering the relationship between objects is beneficial to enhance the understanding of the scene, thereby enhancing the semantics of detection, and bringing it closer to the way of human thinking, it is an important development direction in the future.
4. Pedestrian detection is a core technical problem in the intelligent driving. The current main solution is to use image information for detection. How to use other sensors such as lidar in intelligent driving to enhance the effect of pedestrian detection is an important research direction in the future.

RETRACTED

## Figures and Tables

**Figure 1:** Number of publications related to pedestrian detection in recent years.

**Figure 2:** The development process of pedestrian detection.

**Figure 3:** Faster RCNN series algorithm framework diagram [44, 55, 56]. (a) RCNN. (b) Fast RCNN. (c) Faster RCNN.

**Figure 4:** Algorithm idea of YOLO detector [65].

**Figure 5:** Framework diagram of YOLOv3.

**Figure 6:** CSPNet structure [74].

**Figure 7:** DetNet structure diagram [87]. (a) Dilated bottleneck. (b) Dilated bottleneck with 1 × 1 conv projection. (c) Original bottleneck.

**Figure 8:** Some example images in (a) Caltech [88], (b) KITTI [89], and (c) CityPersons [90].

**Figure 9:** Congestion and obscuration of pedestrian images.

**Figure 10:** Framework diagram of SDS-RCNN [94].

**Figure 11:** Multiscale pedestrian image.

**Figure 12:** Framework diagram of TridentNet [121].

**Table 1:** Calculation speed of some two-stage algorithms.

Method	Model	Rate (fps)
RCNN [44]	AlexNet	13 (s)
Fast RCNN [55]	VGG	2 (s)
Faster RCNN [56]	VGG	5
Comp ACT [60]	VGG	2.5
RFCN [61]	ResNet	5.9
Mask RCNN [3]	ResNet-FPN	5
FPN [62]	ResNet	5
SAF RCNN [64]	VGG	1.7

**Table 2:** Calculation speed of some one-stage algorithms.

Method	Backbone	Rate (fps)
YOLOv1 [65]	—	45
YOLOv2 [67]	Darknet	40
YOLOv3 [68]	Darknet	34.5
YOLOv4 [73]	Darknet	65
SSD [69]	VGG	59
RetinaNet [70]	ResNet-FPN	13.7
ALFnet [71]	ResNet	3.7

**Table 3:** Dataset related information.

Dataset name	Category	Images of train	Images of test	Size	Characteristic
Caltech	1	192000 (persons)	155000 (persons)	640 × 480	Large amount of data and rich annotation information
KITTI	8	7481	7518	1242 × 375	Capture datasets in rural areas and highways, each image contains up to 15 cars and 30 pedestrians
CityPersons	1	2975	500	2048 × 1024	The training set contains approximately 19,744 pedestrians and the test set contains 11 000 pedestrians
EuroCity	1	47300 (238300 persons)	—	1920 × 1024	Pedestrians and riders are carefully marked; especially posters and portraits are marked separately
TUD	1	1284	250	720 × 576	Evaluate the role of motion information in pedestrian detection and provide image pairs to calculate optical flow information
COCO	80	118000	46000	—	Multiple categories, large-scale datasets

**Table 4:** Overall data.

Methods	Miss rate (%)	Methods	Miss rate (%)
SA-FastRCNN [64]	63	F-DNN	51
PCN [93]	62	F-DNN + SS	50
SDS-RCNN [94]	61	F-DNN2 + SS	50
MS-CNN [95]	61	GDFL	48
AdaptFasterRCNN [90]	60	ADM	42
AR-Ped [96]	59	TLL-TFA	38
FasterRCNN + ATT [97]	55		

**Table 5:** Far scale data.

Methods	Miss rate (%)	Methods	Miss rate (%)
MultiFtr + CSS	97	F-DNN	77
CrossTalk	97	F-dnn + SS	77
AFS + Geo	97	F-DNN2 + SS	76
FeatSynth	96	ADM	75
FPDW	96	GDFL	71
ChnFtrs	95	TLL-TFA	60
FasterRCNN + ATT	91		

**Table 6:** Heavy occlusion data.

Methods	Miss rate (%)	Methods	Miss rate (%)
DeepParts	60	AR-Ped	49
MS-CNN	60	FasterRCNN + ATT	45
SDS-RCNN	59	GDFL	43
AdaptFasterRCNN	58	F-DNN2 + SS	40
PCN	56	ADM	30
F-DNN	55	TLL-TFA	29
F-dnn + SS	54		

RETRACTED

**Table 7:** Pedestrian occlusion ratio in the CityPersons dataset.

Total number of pedestrians	IoU between pedestrians is greater than 0.1 (%)	IoU between pedestrians is greater than 0.3 (%)
3157	48.8	26.4

**Table 8:** Calculation speed of some occlusion problem processing algorithm.

Method	Backbone	Rate (fps)
SDS-RCNN [94]	VGG	5
SSA-CNN [105]	VGG	9.1
Adaptive NMS [106]	VGG	—
RepLoss [107]	ResNet	—
OR-CNN [108]	VGG16	—

**Table 9:** Calculation speed of some multiscale problem processing algorithm.

Method	Backbone	Rate (fps)
MCF [110]	VGG	0.54 (CPU)
HyperLearner [111]	VGG	7.1
CFM [112]	VGG	0.8
TLL [113]	ResNet	—
MS-CNN [95]	VGG	15
TridentNet [121]	ResNet	—

## References

[1] Hariharan B., Arbelaez P., Girshick R. Simultaneous detection and segmentation.

[2] Dai J., He K., Sun J. Instance-aware semantic segmentation via multi-task network cascades.

[3] He K., Gkioxari G., Dollar P. Mask r-cnn.

[4] Kang K., Li H., Yan J. (2018). T-cnn: tubelets with convolutional neural networks for object detection from videos. *IEEE Transactions on Circuits and Systems for Video Technology*.

[5] Li M., Xie Q., Zhao Q. Video rain streak removal by multiscale convolutional sparse coding.

[6] Wei W., Meng D., Zhao Q. Semi-supervised transfer learning for image rain removal.

[7] Li Y., Liang R., Wei W. (2021). Temporal pyramid network with spatial-temporal attention for pedestrian trajectory prediction. *IEEE Transactions on Network Science and Engineering*.

[8] Ye D., Zhou B., Zhong B. POCS-based super-resolution image reconstruction using local gradient constraint.

[9] Zhou B., Ye D., Wei W. (2020). Alternating direction projections onto convex sets for super-resolution image reconstruction. *Information Technology and Control*.

[10] Wei W., Yang X., Zhou B. (2012). Combined energy minimization for image reconstruction from few views. *Mathematical Problems In Engineering*.

[11] Li L., Yang M., Guo L. (2017). Precise and reliable localization of intelligent vehicles for safe driving. *Intelligent Autonomous Systems*.

[12] Premebida C., Ludwig O., Nunes U. Exploiting LIDAR-based features on pedestrian detection in urban scenarios.

[13] Jo K., Lee S., Kim C. (2019). Rapid motion segmentation of LiDAR point cloud based on a combination of probabilistic and evidential approaches for intelligent vehicles. *Sensors*.

[14] Wei W., Song H., Li W. (2017). Gradient-driven parking navigation using a continuous information potential field based on wireless sensor network. *Information Sciences*.

RETRACTED

[15] Sun Z., Zhang Y., Nie Y. (2017). CASMOC: a novel complex alliance strategy with multi-objective optimization of coverage in wireless sensor networks. *Wireless Networks*.

[16] Sun Z., Wu W., Wang H. (2014). An optimized strategy coverage control algorithm for WSN. *International Journal of Distributed Sensor Networks*.

[17] Qiang Y., Pei B., Wei W. (2015). An efficient cluster head selection approach for collaborative data processing in wireless sensor networks. *International Journal of Distributed Sensor Networks*.

[18] Fan X., Wei W., Wozniak M. (2018). Low energy consumption and data redundancy approach of wireless sensor networks with bigdata. *Information Technology and Control*.

[19] Li W., Santos I., Delicato F. (2017). System modelling and performance evaluation of a three-tier Cloud of Things. *Future Generation Computer Systems-The International Journal of Escience*.

[20] Chen S., Chiang D., Liu C. (2016). Confidentiality protection of digital health records in cloud computing. *Journal of Medical Systems*.

[21] Liu Y., Sun X., Wei W. (2018). Enhancing energy-efficient and QoS dynamic virtual machine consolidation method in cloud environment. *IEEE Access*.

[22] Wei W., Fan X., Song H. (2018). Imperfect information dynamic stackelberg game based resource allocation using hidden Markov for cloud computing. *IEEE Transactions On Services Computing*.

[23] Qi S., Lu Y., Wei W. (2021). Efficient data access control with fine-grained data protection in cloud-assisted IIoT. *IEEE Internet of Things Journal*.

[24] Liu L., Ouyang W., Wang X. (2018). Deep learning for generic object detection: a survey. *International Journal of Computer Vision*.

[25] Agarwal S., Terrail J. O. D., Jurie F. (2018). Recent advances in object detection in the age of deep convolutional neural networks. http://arxiv.org/abs/1809.03193.

[26] Huang J., Rathod V., Sun C. Speed/accuracy trade-offs for modern convolutional object detectors.

[27] Zou Z., Shi Z., Guo Y. (2019). *Object Detection in 20 Years: A Survey*.

[28] Xiao Y., Zhou K., Cui G. (2021). Deep learning for occluded and multi-scale pedestrian detection: a review. *Iet Image Processing*.

[29] Viola P., Jones M. Rapid object detection using a boosted cascade of simple features.

[30] Dalal N., Triggs B. Histograms of oriented gradients for human detection.

[31] Felzenszwalb P., McAllester D., Ramanan D. A discriminatively trained, multiscale, deformable part model.

[32] Zhou B., Duan X., Wei W. (2019). An adaptive local descriptor embedding zernike moments for image matching. *IEEE Access*.

[33] Zhou B., Duan X., Ye D. (2019). Heterogeneous image matching via a novel feature describing model. *Applied Sciences-Basel*.

RETRACTED

[34] Ge H., Zhu Z., Lou K. (2020). Classification of infrared objects in manifold space using kullback-leibler divergence of Gaussian distributions of image points. *Symmetry-basel*.

[35] Zhao J., Jin W., Wei W. (2013). Enhanced boundary detection method based on Canny theory. *Information Technology Journal*.

[36] Ke Q., Sun Z., Liu Y. (2020). High-resolution sar image despeckling based on nonlocal means filter and modified AA model. *Security and Communication Networks*.

[37] Zhang Y., Wei W., Yuan Y. (2019). Multi-focus image fusion with alternating guided filtering. *Signal Image and Video Processing*.

[38] Ke Q., Zhang J., Song H. (2018). Big data analytics enabled by feature extraction based on partial independence. *Neurocomputing*.

[39] Zhou B., Duan X., Ye D. (2019). Multi-level features extraction for discontinuous target tracking in remote sensing image monitoring. *Sensors*.

[40] Wei W., Li X., Liu J. Study on remote sensing image vegetation classification method based on decision tree classifier.

[41] Zhang L., Shen P., Peng X. (2016). Simultaneous enhancement and noise reduction of a single low-light image. *IET Image Processing*.

[42] Wei W., Zhou B. (2012). A p-laplace equation model for image denoising. *Information Technology Journal*.

[43] Wei W., Sun Z., Zhang Z. (2021). Improved Fisher MAP filter for despeckling of high-resolution SAR images based on structural information detection. *Journal of Internet Technology*.

[44] Girshick R., Donahue J., Darrell T. Rich feature hierarchies for accurate object detection and semantic segmentation.

[45] Wei W., Zhou B., Maskeliunas R. (2019). Iterative design and implementation of rapid gradient descent method. *Artificial Intelligenceand Soft Computing*.

[46] Polap D., Wozniak M., Wei W. (2018). Multi-threaded learning control mechanism for neural networks. *Future Generation Computer Systems-The International Journal of Escience*.

[47] Zhou M., Bai Z., Yi T. (2020). Performance predict method based on neural architecture search. *Journal of Internet Technology*.

[48] Zhang M., Jing W., Lin J. (2020). Automatic design and architecture search of neural network for semantic segmentation in remote sensing images. *Sensors*.

[49] Chen G., Li C., Wei W., Blazauskas T., Damasevicius R. (2019). Fully convolutional neural network with augmented atrous spatial pyramid pool and fully connected fusion path for high resolution remote sensing image segmentation. *Applied Sciences-Basel*.

[50] Wang C., Wei W., Zhang J. (2018). Robust face recognition via discriminative and common hybrid dictionary learning. *Applied Intelligence*.

[51] Shen P., Zhang L., Song J. (2014). A near-infrared face detection and recognition system using ASM and PCA+LDA. *Journal of Networks*.

RETRACTED

[52] Yang F., Qiao Y., Wei W. (2020). DDTree: a hybrid deep learning model for real-time waterway depth prediction and smart navigation. *Applied Sciences-Basel*.

[53] Hu H., Tang B., Gong X. (2017). Intelligent fault diagnosis of the high-speed train with big data based on deep neural networks. *IEEE Transactions On Industrial Informatics*.

[54] Van de Sande K. E., Uijlings J. R., Gevers T. Segmentation as selective search for object recognition.

[55] Girshick R. Fast r-cnn.

[56] Ren S., He K., Girshick R. (2015). Faster R-CNN: towards real-time object detection with region proposal networks. *Advances in Neural Information Processing Systems*.

[57] Everingham M., Van Gool L., Williams C. K. (2010). The pascal visual object classes (voc) challenge. *International Journal of Computer Vision*.

[58] Everingham M., Eslami S. A., Van Gool L. (2015). The pascal visual object classes challenge: a retrospective. *International Journal of Computer Vision*.

[59] Lin T.-Y., Maire M., Belongie S. Microsoft coco: common objects in context.

[60] Cai Z., Saberianet M., Vasconcelosa N. Learning complexity-aware cascades for deep pedestrian detection.

[61] Dai J., Li Y., He K. (2016). Object detection via region-based fully convolutional networks. *Advances in Neural Information Processing Systems*.

[62] Lin T.-Y., Dollar P., Girshick R. B. Feature pyramid networks for object detection.

[63] Divvala S. K., Hoiem D., Hays J. H. An empirical study of context in object detection.

[64] Li J., Liang X., Shen S. (2018). Scale-Aware fast R-CNN for pedestrian detection. *IEEE Transactions on Multimedia*.

[65] Redmon J., Divvala S., Girshick R. You only look once: unified, real-time object detection.

[66] Wu B., Iandola F. N., Jin P. H. Squeezedet: unified, small, low power fully convolutional neural networks for real-time object detection for autonomous driving.

[67] Redmon J., Farhadi A. Yolo9000: better, faster, stronger.

[68] Redmon J., Farhadi A. (2018). Yolov3: an incremental improvement. http://arxiv.org/abs/1804.02767.

[69] Liu W., Anguelov D., Erhan D. Ssd: single shot multibox detector.

[70] Lin T.-Y., Goyal P., Girshick R. (2018). Focal loss for dense object detection. *IEEE Transactions On Pattern Analysis And Machine Intelligence*.

[71] Liu W., Liao S., Hu W. Learning efficient single-stage pedestrian detectors by asymptotic localization fitting.

[72] Zheng Z., Wang P., Liu W. (2019). *Distance-IoU Loss: Faster and Better Learning for Bounding Box Regression*.

[73] Wang B. A., Liao C. W. (2020). *Optimal Speed and Accuracy of Object Detection*.

RETRACTED

[74] Wang C., Liao H., Wu Y. CSPNet: a new backbone that can enhance learning capability of CNN.

[75] He K., Zhang X., Ren S. (2015). Spatial pyramid pooling in deep convolutional networks for visual recognition. *IEEE Transactions on Pattern Analysis and Machine Intelligence*.

[76] Liu S., Qi L., Qin H. Path aggregation network for instance segmentation.

[77] Dong S., Shan Z., Wei W. Visual clustering methods with feature displayed function for self-organizing.

[78] Zhang L., Wei L., Shen P. (2018). Semantic SLAM based on object detection and improved octomap. *IEEE Access*.

[79] Krizhevsky A., Sutskever I., Hinton G. E. (2012). Imagenet classification with deep convolutional neural networks. *Advances in Neural Information Processing Systems*.

[80] Simonyan K., Zisserman A. (2014). Very deep convolutional networks for large-scale image recognition. http://arxiv.org/abs/1409.1556.

[81] Szegedy C., Vanhoucke V., Ioffe S. Rethinking the inception architecture for computer vision.

[82] Szegedy C., Liu W., Jia Y. Going deeper with convolutions.

[83] Ioffe S., Szegedy C. (2015). Batch normalization: accelerating deep network training by reducing internal covariate shift. http://arxiv.org/abs/1502.03167.

[84] Szegedy C., Ioffe S., Vanhoucke V. Inception-v4, inception-resnet and the impact of residual connections on learning.

[85] He K., Zhang X., Ren S. Deep residual learning for image recognition.

[86] Huang G., Liu Z., Van Der Maaten L. (2017). Densely connected convolutional networks. *ICVPR*.

[87] Li Z., Peng C., Yu G. (2018). Detnet: a backbone network for object detection. http://arxiv.org/abs/1804.06215.

[88] Dollar P., Wojek C., Schiele B. (2012). Pedestrian detection: an evaluation of the state of the art. *IEEE Transactions on Pattern Analysis and Machine Intelligence*.

[89] Geiger A., Lenz P., Urtasun R. Are we ready for autonomous driving? the KITTI vision benchmark suite.

[90] Zhang S., Benenson R., Schiele B. (2017). A diverse dataset for pedestrian detection. *Computer Vision And Pattern Recognition*.

[91] Ess A., Leibe B., Van Gool L. Depth and appearance for mobile scene analysis.

[92] Braun M., Krebs S., Flohr F. (2018). The eurocity persons dataset: a novel benchmark for object detection. http://arxiv.org/abs/1805.07193.

[93] Shi X., Shan S., Kan M. Real-time rotation-invariant face detection with progressive calibration networks.

[94] Brazil G., Yin X., Liu X. Illuminating pedestrians via simultaneous detection & segmentation.

[95] Cai Z., Fan Q., S F. R. A unified multi‐scale deep convolutional neural network for fast object detection.

[96] Perez D., Hasan M., Shen Y. (2019). A framework of augmented reality enabled pedestrian-in-the-loop simulation. *Simulation Modelling Practice and Theory*.

RETRACTED

[97] Zhang S., Yang J., Schiele B. Occluded pedestrian detection through guided attention in CNNs.

[98] Wang X., Shrivastava A., Gupta A. A-fast-rcnn: hard positive generation via adversary for object detection.

[99] Mohan A., Papageorgiou C., Poggio T. (2001). Examplebased object detection in images by components. *IEEE Transactions on Pattern Analysis & Machine Intelligence*.

[100] Wu B., Nevatia R. Detection of multiple, partially occluded humans in a single image by bayesian combination of edgelet part detectors.

[101] Wang X., Han T. X. An hog-lbp human detector with partial occlusion handling.

[102] Ouyang W., Wang X. Joint deep learning for pedestrian detection.

[103] Zhou C. Learning to integrate occlusion-specific detectors for heavily occluded pedestrian detection.

[104] Liu L., Wei W., Li X. (2016). Visual attention model based on particle filter. *Ksii Transactions On Internet and Information Systems*.

[105] Zhou C., Wu M., Lam S. Semantic self-attention CNN for pedestrian Detection.

[106] Liu S., Huang D., Wang Y. (2019). Adaptive NMS: refining pedestrian detection in a crowd. http://arxiv.org/abs/1904.03629.

[107] Wang X., Xiao T., Jiang Y. Repulsion loss: detecting pedestrians in a crowd.

[108] Zhang S., Wen L., Bian X. Occlusion-aware R-CNN: detecting pedestrians in a crowd.

[109] Wang X., Han T. X., Yan S. An hog-lbp human detector with partial occlusion handling.

[110] Cao J., Pang Y., Li X. (2017). Learning multilayer channel features for pedestrian detection. *IEEE Transactions on Image Processing*.

[111] Mao J., Xiao T., Jiang Y. What can help pedestrian detection?.

[112] Hu Q., Wang P., Shen C. (2018). Pushing the limits of deep cnns for pedestrian detection. *IEEE Transactions on Circuits and Systems for Video Technology*.

[113] Song T., Sun L., Xie D. Small-scale pedestrian detection based on somatic topology localization and temporal feature aggregation.

[114] Zhang S., Benenson R., Omran M. How far are we from solving pedestrian detection?.

[115] Qin J., Yung N. H. (2012). Feature fusion within local region using localized maximum-margin learning for scene categorization. *Pattern Recognition*.

[116] Zhou P., Ni B., Geng C. Scaletransferrable object detection.

[117] Jeong J., Park H., Kwak N. (2017). Enhancement of Ssd by concatenating feature maps for object detection. http://arxiv.org/abs/1705.09587.

[118] Lee K., Choi J., Jeong J. (2017). Residual features and unified prediction network for single stage detection. http://arxiv.org/abs/1707.05031.

[119] Shrivastava A., Sukthankar R., Malik J. (2016). Beyond skip connections: top-down modulation for object detection. http://arxiv.org/abs1612.06851.

RETRACTED

[120] Woo S., Hwang S., Kweon I. S. Top-down semantic aggregation for accurate one shot detection.

[121] Li Y., Chen Y., Wang N. Scale-Aware trident networks for object detection.

[122] Voulodimos A., Doulamis N., Doulamis A. (2018). Deep learning for computer vision: a brief review. *Computational Intelligence and Neuroscience*.

[123] Guo Y., Liu Y., Oerlemans A. (2016). Deep learning for visual understanding: a review. *Neurocomputing*.

[124] Hurney P., Waldron P., Morgan F. (2015). Review of pedestrian detection techniques in automotive far-infrared video. *IET Intelligent Transport Systems*.

[125] Benenson R., Omran M., Hosang J. Ten years of pedestrian detection, what have we learned?.

[126] Geronimo D., Lopez A., Sappa A. (2014). Survey of pedestrian detection for advanced driver assistance systems. *IEEE Transactions on Pattern Analysis and Machine Intelligence*.

[127] Sumit S., Rambli D., Mirjalili S. (2021). Vision-based human detection techniques: a descriptive review. *IEEE Access*.

